# Clinicopathological, Oncogenic, and ^18^F-FDG PET/CT Features of Primary Pulmonary Carcinoid in Resection Specimens

**DOI:** 10.1155/2022/1926797

**Published:** 2022-06-15

**Authors:** Yun Chen, Yun Dong, Jingyun Shi, Long Zhao

**Affiliations:** ^1^Department of Radiation Oncology, Shanghai Pulmonary Hospital, School of Medicine, Tongji University, Shanghai 200092, China; ^2^Department of Radiation Oncology, No. 9 People Hospital Affiliated to Shanghai JiaoTong University School of Medicine, Shanghai 201999, China; ^3^Department of Radioology, Shanghai Pulmonary Hospital, School of Medicine, Tongji University, Shanghai 200092, China; ^4^Department of Nuclear Medicine, Shanghai Pulmonary Hospital, School of Medicine, Tongji University, Shanghai 200092, China

## Abstract

**Objectives:**

The metabolic parameters which included mean standardised uptake value (SUVmean), metabolic tumour volume (MTV), total lesion glycolysis (TLG), maximum standardised uptake lean body mass (SULmax), and maximum standardised uptake body surface area (SUVbsa) have rarely been investigated in pulmonary carcinoid (PC). This study aimed to retrospectively compare the ^18^F-FDG PET/CT features of PC subtypes and observe clinicopathological and oncogenic characteristics of PC.

**Methods:**

We performed a retrospective review in 60 patients with PC, from January 2016 to November 2021, who underwent the ^18^F-FDG PET/CT scan. All the PC diagnoses were histopathologic confirmed by surgical samples. The metabolic and morphological features were obtained from ^18^F-FDG PET/CT images. The ratio of metabolic to morphological lesion volumes (MMVR) was calculated.

**Results:**

Sixty patients with PC were consecutively identified, including 39 patients (65.0%) with typical carcinoids (TCs) and 21 (35.0%) with atypical carcinoids (ACs). One (1/21) patient had mutation in BRAF. The ACs have a larger size (*P* < 0.001), more metastatic lymph nodes (*P* = 0.011), higher Ki-67 expression (*P* < 0.001), higher SUVmax values (*P* = 0.003), higher SUVmean values (*P* = 0.006), higher SULmax values (*P* = 0.005), higher SUVbsa values (*P* = 0.001), higher MTV values (*P* = 0.033), and higher TLG values (*P* = 0.002). The multivariate analysis showed that MMVR (*P* = 0.020) was significantly associated with AC. For predicting AC, the optimal cut-off value of SUVmax, SUVmean, SULmax, SUVbsa, MTV, TLG, and the maximum diameter was 5.19, 3.18, 2.65, 1.47, 4.36, 18.44, and 3.0, respectively. The AUC values of above mentioned parameters was 0.756 (95%CI, 0.631–881; *P* = 0.001), 0.735 (95%CI, 0.602–868; *P* = 0.003), 0.736 (95%CI, 0.607–865; *P* = 0.003), 0.742 (95%CI, 0.612–873; *P* = 0.002), 0.593 (95%CI, 0.430–755; *P* = 0.239), 0.680 (95%CI, 0.531–829; *P* = 0.022), and 0.733 (95%CI, 0.598–868; *P* = 0.003), respectively. For predicting TC, the optimal cut-off value of the MMVR was 0.92, and the AUC value was 0.780 (95%CI, 0.647–0.913; *P* < 0.001).

**Conclusion:**

^18^F-FDG PET/CT can simultaneously reveal the metabolic and morphological characteristics of PC, which is important in the differentiation for histopathologic subtypes.

## 1. Introduction

Pulmonary carcinoid (PC) tumors are a rare subtype of neuroendocrine malignancies, accounting for less than 2% of all lung malignancies [1, 2]. Environmental risk factors, including harmful maternal exposures, have yet to be identified for PC although tobacco smoking has been proposed [3]. Patients often present with nonspecific symptoms including cough, wheezing, dyspnea, chest pain, haemoptysis, and chronic obstructive pulmonary disease. In addition, patients with Cushing disease can occasionally present with flushing, palpitations, abdominal pain, and diarrhea [4]. However, these symptoms are considered insufficiently specific to diagnose PC on their own. In fact, as PC often manifests as a localized slowly growing mass, the majority of patients have no symptoms at all and are more likely to be diagnosed incidentally during investigation of a separate medical issue.

PCs are thought to originate from enterochromaffin (Kulchitsky) cells in the bronchial and bronchiolar mucosa. PC tumors can be subdivided into two categories according to the mitotic rate and the presence or absence of necrosis. Typical carcinoids (TCs) are well differentiated, of low-grade (less than two mitoses per 2 mm^2^ and lack of necrosis), and less aggressive [5]. Atypical carcinoids (ACs) are poorly differentiated, of intermediate-grade (more than two mitoses per 2 mm^2^, and necrosis may be present), and more likely to exhibit regional lymph node or distant metastases [5]. Complete surgical resection is the therapeutic option that offers the best prognosis for patients. The surgical treatment regimen depends on the size, location, and histological subtype; the goal of surgery is to preserve as much lung tissue as possible while still eliminating the tumor. Thus, preoperative differentiation of TC and AC is critical for designing surgical plans and predicting prognosis.

Positron emission tomography (PET), using different tracers, has been used to differentiate between ACs and TCs. The maximum standardised uptake (SUV_max_) of ^18^-fluoro-deoxyglucose (^18^FDG) and ^68^Ga-DOTA-labeled somatostatin analogues likely has limited value in the differential diagnosis of histological subtype [6–11]. ^18^FDG SUV_max_ values are higher in AC than in TC, whereas ^68^Ga-DOTA-labeled somatostatin analogues SUV_max_ values were higher in TC than in AC. These studies also showed that the ratio of SUV_max_ of ^68^Ga-DOTA-labeled somatostatin analogues to that of ^18^FDG provided the best diagnostic performance for predicting the histopathologic variety of PC. However, unfortunately, ^68^Ga-DOTA-labeled somatostatin analogues are only available in a limited number of hospitals in China. Moreover, other metabolic parameters, including mean SUV (SUV_mean_), metabolic tumor volume (MTV), total lesion glycolysis (TLG), maximum standardised uptake lean body mass (SUL_max_), and maximum standardised uptake body surface area (SUVbsa) between PC subtypes have rarely been reported. Thus, the goals of this study were to retrospectively compare the ^18^F-FDG PET/CT features of PC subtypes and observe clinicopathological and oncogenic characteristics of PC.

## 2. Materials and Methods

### 2.1. Study Population

We performed a retrospective review of patients who underwent PET/CT by searching our hospital's database for relevant cases occurring between January 2016 and November 2021(Figure 1). This study was approved by the institutional review board of our hospital. Sixty patients with PC were enrolled based on the following criteria: (1) newly diagnosed with PC and histopathological results confirmed via surgical pathological examination, (2) no previous history of malignancy, (3) no antitumor treatment before PET/CT scanning and surgery, (4) an interval between PET/CT scanning and surgery of less than one month, and (5) lesions were measurable and were clearly delineated. Clinicopathological characteristics of each patient were retrospectively obtained from electronic medical records.

### 2.2. ^18^F–FDG PET/CT Scanning and Analysis

^18^F-FDG PET/CT imaging was performed using a PET/CT scanner (Biograph Mct64, Siemens, Erlangen, Germany). Patients with both a fasting (4–6 h) and serum glucose level <11.1 nmol/L were injected with 0.10–0.15 mCi/kg of ^18^F-FDG. All patients rested for an hour and then underwent whole-body PET/CT scanning (six or seven bed positions from upper thighs to forehead) according to the manufacturer's protocol. All patients also underwent an additional thin-section, chest CT scan at full inspiration with a slice thickness of 1 mm. Two independent experienced nuclear medicine physicians (Z.L., L.Q.), blinded to the clinicopathological information, retrospectively performed metabolic parameter measurements and a morphological feature assessment of the primary tumor. Metabolic parameters included SUV_max_, SUV_mean_, SUL_max_, SUVbsa, MTV, and TLG (TLG = MTV × SUVmean). Using a threshold of 40% of the SUVmax by an SUV-based automated contouring program, the contour of the primary tumor was defined on attenuation-corrected ^18^F-FDG PET/CT images.

The ratio of metabolic to morphological lesion volumes (MMVR) was calculated (MMVR = MTV/morphological tumour volume). Morphological tumour volume was calculated based on the modified ellipsoidal formula on CT images. The morphological features included (1) size (maximum diameter of the primary lesion), (2) location (central or peripheral), (3) mass attenuation by CT (HU), (4) marginal characteristics (lobulated border and spiculation), (5) pleural characteristics (pleural indentation and pleural effusion), (6) bronchiectasis, (7) atelectasis, (8) calcifications, (9) airway involvement, and (10) opacity around the lesion.

### 2.3. Immunohistochemistry and Mutational Analyses

Tumor samples were obtained by surgical resection. All resected tissues were subject to formalin fixation, paraffin embedding, and immunohistochemical stains following standard procedures of the Department of Pathology in our hospital. Immunohistochemical staining for differentiation markers including CD56, chromogranin A (CgA), synaptophysin (Syn), thyroid transcription factor 1 (TTF-1), S-100, INSM1, and Ki-67 was conducted. Aberrations of the epidermal growth factor receptor (*EGFR*) (exons 18–22), Kirsten rat sarcoma viral oncogene homolog (*KRAS*) (exons 2–3), B-type Raf kinase (*BRAF*), echinoderm microtubule-associated protein-like 4-anaplastic lymphoma kinase (*EML4-ALK*), and C-ros oncogene 1 (*ROS1*) were measured. The status of driver gene mutations was assessed according to standard clinical operating procedures.

### 2.4. Statistics

Patient characteristics are descriptively summarized using the mean ± SD or frequencies (percentages) for continuous and categorical variables, respectively. Pathological features as well as metabolic and morphological parameters are also described, as appropriate. Features were compared between patients with AC versus TC using either a *χ*^2^ test or Mann–Whitney *U* test. To predict the presence of AC or TC, receiver operating characteristic (ROC) analysis was employed to calculate optimal cut-off values; the sensitivity, specificity, positive-predictive value, negative-predictive value, accuracy, and the area under the curve (AUC) were also calculated for each variable. Differences were considered statistically significant when *P* < 0.05. Data in this study were statistically analyzed using a software program (version 21.0; IBM, Armonk, NY, USA).

## 3. Results

### 3.1. Clinicopathological Findings

Clinical characteristics of all patients are summarized in Table 1. A total of 60 patients were included, of which 25 (41.7%) were males and 35 were females (58.3%). The mean age of all patients was 54.1 ± 13.3 years (22–82); the mean age of patients with TC was 54.7 ± 11.1 years and the mean age of patients with AC was 53.1 ± 16.8 years . Twenty-one (35.0%) smokers and 39 (65.0%) nonsmokers were included in this study. Twenty-one (35.0%) patients with AC and 39 (65.0%) patients with TC underwent surgical resection of their tumor. Twenty-nine patients (48.3%) with PC presented with symptoms, of which 25 patients complained of cough; of the 25 patients with cough, ten presented with haemoptysis. Two patients complained of dyspnea, and two patients exhibited fever. In addition, AC patients had a significantly greater number of metastatic lymph nodes than patients with TC (8/72.7% vs 3/27.3%, *P* = 0.011).

### 3.2. Immunohistochemistry and Gene Expression Findings 

Immunohistochemistry was used to assess the expression of CD56, TTF-1, Syn, CgA, INSM1, Ki-67, and S-100 in resected tumor tissue samples; detailed information is presented in Table 2. In this study, proliferation marker Ki-67 expression was higher in patients with AC than that in patients with TC (*P* < 0.001). TTF-1 tended to be positive in peripheral tumors but negative in central tumors (51.6% vs. 14.3%, *P* = 0.003), and the result was not shown. Mutations in *EGFR*, *EML4-ALK*, and *ROS1* were evaluated in 36 patients; however, no mutations were detected. The mutation status of *KRAS* and *BRAF* was evaluated in 21 patients; one patient had mutation in *BRAF*.

### 3.3. ^18^F-FDG PET/CT Findings

Metabolic and morphological features of tumor tissue from patients with PC were assessed using ^18^F-FDG PET/CT scans and are summarized in Table 3. The mean maximum diameter of PC tumors was 2.2 ± 1.3 cm (ranging, 0.6–7.0 cm), while the median maximum diameter of TC tumors was 1.8 cm (interquartile range, 1.3–2.8 cm). AC tumors thus had larger diameters than TC tumors (*P* < 0.001). No other radiological differences were identified between AC and TC tumors.

Metabolic parameters, including median values (interquartile range) of SUV_max_, SUV_mean_, SUL_max_, SUVbsa, MTV, and TLG are listed in Table 3. The mean values of SUV_max_, SUV_mean_, SUL_max_, SUVbsa, MTV, and TLG were 5.65 ± 7.45, 3.51 ± 4.98, 5.33 ± 7.96, 1.66 ± 2.33, 8.09 ± 13.78, and 30.72 ± 63.38, respectively. Results of Mann–Whitney *U* test are also shown in Figure 2. PET parameters of the median SUV_max_ (*P* = 0.003), SUV_mean_ (*P* = 0.006), SUL_max_ (*P* = 0.005), SUVbsa (*P* = 0.002), MTV (*P* = 0.033), and TLG (*P* = 0.002) were lower in TC tumors than in AC tumors (Figure 2).  Figure 3 shows AC tumors had lower MMVR values (*P* < 0.001). However, the multivariate analysis showed that only MMVR (*P* = 0.020) was significantly associated with AC (Table 4). For predicting AC, the optimal cut-off value of SUVmax, SUVmean, SULmax, SUVbsa, MTV, TLG, and maximum diameter was 5.19, 3.18, 2.65, 1.47, 4.36, 18.44, and 3.0, respectively. The AUC values of above mentioned parameters was 0.756 (95%CI, 0.631–881; *P* = 0.001), 0.735 (95%CI, 0.602–868; *P* = 0.003), 0.736 (95%CI, 0.607–865; *P* = 0.003), 0.742 (95%CI, 0.612–873; *P* = 0.002), 0.593 (95%CI, 0.430–755; *P* = 0.239), 0.680 (95%CI, 0.531–829; *P* = 0.022), and 0.733 (95%CI, 0.598–868; *P* = 0.003), respectively (Figure 4). Diagnostic performance for each of the following parameters is listed in Table 5: maximum diameter, SUV_max_, SUV_mean_, SUL_max_, SUVbsa, MTV, and TLG. For predicting TC, the optimal cut-off value of the MMVR was 0.92, and the AUC value was 0.780 (95%CI, 0.647–0.913; *P* < 0.001) (Figure 3).

## 4. Discussion

Pulmonary carcinoids are a rare and heterogeneous group, comprising TC and AC tumor types; prognosis varies with different histological subtypes. However, there is no clear clinical picture that can differentiate between TC and AC tumor types as patients with either type can present asymptomatically or with nonspecific symptoms [4]. Thus, there is a lack of professional consensus regarding diagnostic assessment and treatment options for PC. In this study, use of ^18^F-FDG PET/CT scans revealed a statistically significant difference in several metabolic parameters between TC and AC tumor types.

Clinical findings in patients with PC investigated in this study were consistent with the previously published studies [2, 5, 12, 13]. In our cohort, the mean age was 54.1 years, which also agrees with data previously reported. Petursdottir et al. and Georgakopoulou et al. reported that patients with AC tumors were older than patients with TC tumors, whereas Li et al. and Thakur et al. reported that there were no significant differences between patients with either tissue type [2, 5, 12, 13]. The latter observations are consistent with the results in our study. We report that 48.3% of patients were symptomatic, which differs from the results reported by Petursdottir et al. in which 70.5% of patients were symptomatic. However, the patient cohort in the Petursdottir et al. study comprised a majority of patients (73.9%) with central PC, while our cohort included only 48.3%. Previous studies have indicated that central tumors often present with symptoms related to segmental or larger airway obstruction, while peripheral tumors generally present asymptomatically or are only incidentally detected upon chest imaging [14]. These differences might account for the discrepancy between the results of our study and those of Petursdottir et al.

Our study also found that lymph node metastases were more frequent in patients with AC tumors than in patients with TC tumors (8/72.7% vs 3/27.3%, *P* = 0.011), which was consistent with previous study results [2, 5, 12, 13]. Georgakopoulou et al. reported that patients with surgically-resected pulmonary carcinoids without distant metastases had increased survival [12]. Thakur et al. also reported that the presence and location of lymph node metastases were significant prognostic factors [5]. Thus, it is critical to evaluate preoperative lymph node status when making decisions regarding the extent of surgery.

To the best of our knowledge, cancer-related gene mutations are not common in patients with PC. The low frequency mutations of *EGFR*, *EML4-ALK*, *BRAF*, *KRAS*, *SMAD4*, and *PIK3CA* have previously been reported for PC tumors [15–18]. We only identified a single patient with a *BRAF* mutation in this study. Chen et al. reported that a 72-year-old man with pulmonary atypical carcinoid harbored the *EGFR* L858R mutation [17]. After receiving combination chemotherapy consisting of irinotecan and icotinib plus cisplatin, the patient exhibited a partial response prior to resection. With the advent of precision medicine and the rising attention given to molecular pathology, mutation detection has gradually become the standard of care in clinical practice. It can be expected that patients with rare tumors will also benefit from more personalized treatment. Very little information is known about the genetic background of PCs. Further studies are necessary to validate these results and enhance understanding of their molecular characteristics.

Our immunohistochemical results were similar to those reported by others [19–21]. PC exhibited strong protein expression of neuroendocrine markers such as CD56, Syn, CgA, and INSM1. In addition, TTF-1 positivity was observed at greater frequency in peripheral tumors as compared to central tumors. Our study also revealed that PC tumors with a Ki-67 index ≥5% were more likely to be of the AC subtype. The finding showed that AC tumours exhibited a stronger proliferation activity than TC tumours, which was in line with the former being clinically more aggressive forms. And, the proliferative activity of AC tumors also likely reflects increased mitotic activity. Boland et al. reported that a Ki-67 index ≥3.5% predicted atypical histology for both biopsy and resection [22]. Thus, it may be useful to integrate the Ki-67 index into differential diagnosis of AC tumors and TC tumors. Previous studies have reported that the Ki-67 index is also associated with recurrence and prognosis, but that the cut-off value differs in these studies [19–21]. Further research regarding gene expression in PC is required in order to improve preoperative determination of histological subtype, risk stratification, and prediction of prognosis.

Preoperative evaluation of PC is preferably evaluated via a CT scan. Previous studies have reported that PC often presents with no specific radiographic features, while a lobulated border and direct and indirect findings related to bronchial obstruction are more common [23, 24]. The imaging heterogeneity has also not been established between AC and TC tumors, which have similar imaging characteristics. In this study, AC patients exhibited larger tumor sizes; however, this was not sufficient to correctly distinguish AC from TC tumors. Recent developments in radiomic methods, machine learning, and artificial intelligence have revolutionized radiology. In order to appropriately distinguish AC and TC tumors, future studies may benefit from these advanced methods.

At present, published studies have reported that ^18^F-FDG and ^68^Ga-DOTA-labeled somatostatin analogues used in PET/CT scanning might have limited value in distinguishing the PC subtype [6–11]. SUV_max_ values of ^18^FDG were higher in AC tumors, while SUV_max_ values of ^68^Ga-DOTA-labeled somatostatin analogues were higher in TC tumors. And several studies showed that ^18^F-FDG PET metabolic parameters were not able to distinguish TC from AC [25]. Furthermore, previous studies reported that the SUV_max_ ratio of ^68^Ga-DOTA-labeled somatostatin analogues and ^18^F-FDG is more accurate for the prediction of histological subtype in PC as compared with the SUV_max_ of ^68^Ga-DOTA-labeled somatostatin analogues or ^18^FDG alone [7–11]. According to a meta-analysis, Jiang et al. reported that the SUV_max_ ratio had 89.3% sensitivity and 100% specificity in distinguishing TC from AC [7]. However, ^68^Ga-DOTA-labeled somatostatin analogs are only available in a limited number of hospitals in China. By comparing metabolic parameters, we found that the TLG had the highest specificity (84.6%), while SUL_max_ had the highest sensitivity (85.7%) and negative-predictive value (87.0%). On the other hand, values of MMVR in AC were significantly lower than those in TC. This is the most probably attributed more necrotic area in AC tumours, which can cause low MTV on ^18^FDG PET/CT images. The MMVR had a specificity of 89.7% and an accuracy of 80.0%. And the multivariate analysis showed that only an MMVR was significantly associated with AC. The MMVR may be better than other metabolic parameters for distinguishing TC from AC. The study showed that AC tumours with stronger proliferation activity have higher relative metabolic activity on ^18^FDG PET/CT examination. However, metabolic parameters obtained via ^18^F-FDG were not as good at differentiating histopathologic variety of PC, individually. When ^68^Ga-DOTA-labeled somatostatin analogues are unavailable, ^18^FDG PET/CT scanning can provide valuable additional information in for preoperative differentiation of AC and TC tumors. In recent years, there have been an increasing number of studies related to texture features in the analysis of PET/CT data. In this regard, further studies are needed to improve predictive performance.

This study has several limitations. First, it is an observational, single-center, retrospective study. Second, only patients who underwent surgical resection were included in this study. Both of these limitations can result in selection bias. Finally, the present study did not include contrast enhancement features of CT images in patients with PC because only some patients underwent enhanced CT examination. Moreover, in our hospital, enhanced CT examination were not performed on the same device. The lack of standardization resulted in a lack of uniformity in the data, making them difficult to compare. More rigorous studies are warranted.

## 5. Conclusion

In conclusion, our findings revealed that metabolic parameters of ^18^FDG PET/CT were significantly associated with histopathological subtypes of pulmonary carcinoid. AC tumors tend to be larger and exhibit higher proliferative activity compared with TC tumors. For predicting TC, MMVR is also a valuable option. In the absence of ^68^Ga-DOTA-labeled somatostatin analogues, ^18^FDG PET/CT scanning can assist in preoperative differentiation of AC and TC tumors.

## Figures and Tables

**Figure 1:** Flowchart of the study population.

**Figure 2:** The Mann–Whitney *U* test showed the maximum diameter and most of metabolic parameters of ^18^FDG PET/CT were significantly associated with histological subtypes of pulmonary carcinoid.

**Figure 3:** The ratio of metabolic to morphological lesion volumes (MMVR) were significantly associated with histological subtypes of pulmonary carcinoid. (a) The result of Mann–Whitney *U* test. (b) For predicting TC, the AUC value of MMVR was 0.780 (95%CI, 0.647–0.913; *P* < 0.001). (c) Diagnostic performance parameters.

**Figure 4:** For predicting AC, the AUC values of the SUVmax, SUVmea, SULmax, SUVbsa, MTV, TLG, and maximum diameter was 0.756 (95%CI, 0.631–881; *P* = 0.001), 0.735 (95%CI, 0.602–868; *P* = 0.003), 0.736 (95%CI, 0.607–865; *P* = 0.003), 0.742 (95%CI, 0.612–873; *P* = 0.002), 0.593 (95%CI, 0.430–755; *P* = 0.239), 0.680 (95%CI, 0.531–829; *P* = 0.022), and 0.733 (95%CI, 0.598–868; *P* = 0.003), respectively.

**Table 1:** Baseline characteristics of 60 patients with pulmonary carcinoid.

Clinical factors	Total		Typical carcinoid		Atypical carcinoid		*P* value
	No.	%	No.	%	No.	%	
	60	100.0	39	65.0	21	35.0	
Age (y)	54.1 ± 13.3		54.7 ± 11.1		53.1 ± 16.8		0.703
Sex							0.493
Male	25	41.7	15	60.0	10	40.0	
Female	35	58.3	24	68.6	11	31.4	
Smoking history							0.712
Never	39	65.0	26	66.7	13	33.3	
Former/current	21	35.0	13	61.9	8	38.1	
Symptoms							0.788
Yes	29	48.3	18	62.1	11	37.9	
No	31	51.7	21	67.7	10	32.3	
Site							0.234
LLL	12	20.0	9	75.0	3	25.0	
LUL	10	16.7	4	40.0	6	60.0	
RLL	15	25.0	10	66.7	5	33.3	
RML	15	25.0	12	80.0	3	20.0	
RUL	8	13.3	4	50.0	4	50.0	
Pathological stage							0.058
I	45	75.0	33	73.3	12	26.7	
II	9	15.0	4	44.4	5	55.6	
III	6	10.0	2	33.3	4	66.7	
T stage							0.634
T1	52	86.7	35	67.3	17	32.7	
T2	6	10.0	3	50.0	3	50.0	
T3	2	3.3	1	50.0	1	50.0	
Lymph node metastases							0.011
N0	49	81.7	36	73.5	13	26.5	
N1/N2	11	18.3	3	27.3	8	72.7	

LLL: left lower lobe, LUL: left upper lobe, RLL: right lower lobe, RML: right middle lobe, RUL: right upper lobe.

**Table 2:** Immunohistochemistry results of pulmonary carcinoids.

Clinical factors	Total		Typical carcinoid		Atypical carcinoid		*P* value
	No.	%	No.	%	No.	%	
CD56							0.607
Negative	4	7.0	2	5.4	2	10.0	
Positive	53	93.0	35	94.6	18	90.0	
TTF-1							0.651
Negative	39	66.1	25	64.1	14	70.0	
Positive	20	33.9	14	35.9	6	30.0	
SYN							1.000
Negative	1	1.7	1	2.6	0	0.0	
Positive	58	98.3	38	97.4	20	100.0	
CgA							1.000
Negative	2	9.1	1	12.5	1	0.0	
Positive	56	90.9	38	87.5	18	100.0	
S-100							0.282
Negative	7	46.7	4	36.4	3	75.0	
Positive	8	53.3	7	63.6	1	25.0	
INSM1							0.316
Negative	1	5.3	0	0.0	1	16.7	
Positive	18	94.7	13	100.0	5	83.3	
KI67							<0.001
<5%	44	80.0	35	94.6	9	50.0	
≥5%	11	20.0	2	5.4	9	50.0	

**Table 3:** ^18^F-FDG PET/CT findings of pulmonary carcinoids.

Clinical factors	Total		Typical carcinoid		Atypical carcinoid		*P* value
	No.	%	No.	%	No.	%	
	60	100.0	39	100.0	21	100.0	
Maximum diameter (cm), mean ± SD	2.2 ± 1.3		1.8 ± 0.9		2.9 ± 1.6		0.007
Maximum diameter (cm), median (IQR)	1.8(1.3–2.8)		1.7 (1.1–2.3)		2.7(1.6–3.5)		
<3.0	49	81.7	37	94.9	12	57.1	<0.001
≥3.0	11	18.3	2	5.1	9	42.9	
Mass attenuation on CT (HU) without contrast injection	30.9 ± 17.6		31.5 ± 20.0		29.8 ± 12.6		0.722
Location							0.788
Central	29	48.3	18	46.2	11	52.4	
Peripheral	31	51.7	21	53.8	10	47.6	
Calcification							0.649
No	55	91.7	35	89.7	20	95.2	
Yes	5	8.3	4	10.3	1	4.8	
Lobulated border							0.337
No	35	58.3	21	53.8	14	66.7	
Yes	25	41.7	18	46.2	7	33.3	
Pleural effusion							
No	55	91.7	36	92.3	19	90.5	1
Yes	5	8.3	3	7.7	2	9.5	
Pleural indentation							0.226
No	53	88.3	36	92.3	17	81.0	
Yes	7	11.7	3	7.7	4	19.0	
Spiculated margin							
No	59	98.3	38	97.4	21	100.0	1
Yes	1	1.7	1	2.6	0	0.0	
Airway involvement							
No	20	33.3	13	33.3	7	33.3	1
Yes	40	66.7	26	66.7	14	66.7	
Bronchiectasis							
No	45	75.0	27	69.2	18	85.7	0.16
Yes	15	25.0	12	30.8	3	14.3	
Atelectasis							
No	55	91.7	35	89.7	20	95.2	0.649
Yes	5	8.3	4	10.3	1	4.8	
Opacity							
No	43	71.7	28	71.8	15	71.4	0.976
Yes	17	28.3	11	28.2	6	28.6	
SUVmax (median (IQR))	4.11(2.34–5.87)		3.50 (1.44–5.11)		5.67(4.01–8.33)		0.003
<5.19	38	63.3	30	76.9	8	38.1	
≥5.19	22	36.7	9	23.1	13	61.9	
SUVmean (median (IQR))	2.60 (1.44–3.59)		1.98 (1.18–2.97)		3.22 (2.35–4.82)		0.006
<3.18	42	70.0	32	82.1	10	47.6	
≥3.18	18	30.0	7	17.9	11	52.4	
MTV (median (IQR))	4.16 (2.50–7.32)		3.48(2.49–6.92)		4.80 (2.49–10.62)		0.033
<4.36	34	56.7	26	66.7	8	38.1	
≥4.36	26	43.3	13	33.3	13	61.9	
TLG (median (IQR))	11.10(4.05–21.03)		7.83(3.75–17.01)		18.69 (6.03–88.06)		0.002
<18.44	43	71.7	33	84.6	10	47.6	
≥18.44	17	28.3	6	15.4	11	52.4	
SULmax (median (IQR))	3.81 (2.12–5.53)		2.58 (1.49–4.80)		4.85 (3.30–7.28)		0.005
<2.65	23	38.3	20	51.3	3	14.3	
≥2.65	37	61.7	19	48.7	18	85.7	
SUVbsa (median (IQR))	1.26 (0.66–1.70)		0.81 0.509–1.46)		1.54 (1.03–2.34)		0.001
<1.47	37	61.7	30	76.9	7	33.3	
≥1.47	23	38.3	9	23.1	14	66.7	
MMVR	3.81 (2.12–5.53)		2.58 (1.49–4.80)		4.85 (3.30–7.28)		<0.001
<0.92	17	28.3	4	10.3	13	61.9	
≥0.92	43	71.7	35	89.7	8	38.1	

HU, Hounsfield unit; IQR, interquartile range; MTV, metabolic tumour volume; SULmax, maximum standardised uptake lean body mass; SUVbsa, maximum standardised uptake body surface area; SUVmax, maximum standardised uptake value; SUVmean, mean standard uptake value; TLG, total lesion glycolysis; MMVR, the ratio of metabolic to morphological lesion volumes.

**Table 4:** Multivariate analyses of ^18^F-FDG PET/CT metabolic parameters.

	*P* value	OR	95% CI	
			Lower limit	Upper limit
SUVmax	0.968	0.925	0.021	40.225
SUVmean	0.853	1.310	0.075	22.921
MTV	0.503	1.898	0.291	12.367
TLG	0.533	1.912	0.249	14.652
SULmax	0.755	0.716	0.088	5.847
SUVbsa	0.382	4.035	0.176	92.338
MMVR	0.020	7.531	1.371	41.367

**Table 5:** Diagnostic performance of ^18^F-FDG PET/CT parameters for predicting pulmonary atypical carcinoids.

Parameter	Cut-off value	Sensitivity (%)	Specificity (%)	Positive predictive value (%)	Negative predictive value (%)	Accuracy (%)
Maximum diameter (cm)	3.00	42.9	94.9	81.8	75.5	76.7
SUVmax	5.19	61.9	76.9	59.1	79.0	71.7
SUVmean	3.18	52.4	82.1	61.1	76.2	71.7
MTV	4.36	61.9	66.7	50.0	76.5	65.0
TLG	18.44	52.4	84.6	64.7	76.7	73.3
SULmax	2.65	85.7	51.3	48.7	87.0	63.3
SUVbsa	1.47	66.7	76.9	60.9	81.1	73.3

## Data Availability

The datasets used and/or analyzed during the current study are available from the corresponding author on reasonable request.

## Abbreviations

^18^F-FDG PET/CT: ^18^F-fluorodeoxyglucose positron emission tomography/computed tomography
SUVmax: Maximum standardised uptake value
SULmax: Maximum standardised uptake lean body mass
SUVmean: Mean standard uptake value
SUVbsa: Maximum standardised uptake body surface area
MTV: Metabolic tumour volume
TLG: Total lesion glycolysis
MMVR: The ratio of metabolic to morphological lesion volumes
PC: Pulmonary carcinoid
AC: Atypical carcinoids
TC: Typical carcinoids
EGFR: Epidermal growth factor receptor
KRAS: Kirsten rat sarcoma viral oncogene homolog
BRAF: B-type Raf kinase
EML4-ALK: Echinoderm microtubule-associated protein-like 4-anaplastic lymphoma kinase
ROS1: C-ros oncogene 1.
